The article "A View on Polymerase Chain Reaction as an Outstanding Molecular Diagnostic Technique in Periodontology" was published in 2021. Journal: Biomed Res Int.

# A View on Polymerase Chain Reaction as an Outstanding Molecular Diagnostic Technique in Periodontology

**DOI:** 10.1155/2021/9979948

**Published:** 2021-07-19

**Authors:** Adileh Shirmohammadi, Amirreza Babaloo, Solmaz Maleki Dizaj, Farzaneh Lotfipour, Simin Sharifi, Mohammad Ali Ghavimi, Khadijeh Khezri

**Affiliations:** ^1^Department of Periodontics, Faculty of Dentistry, Tabriz University of Medical Sciences, Tabriz, Iran; ^2^Dental and Periodontal Research Center, Tabriz University of Medical Sciences, Tabriz, Iran; ^3^Department of Dental Biomaterials, Faculty of Dentistry, Tabriz University of Medical Sciences, Tabriz, Iran; ^4^Food and Drug Safety Research Center, Tabriz University of Medical Sciences, Tabriz, Iran; ^5^Faculty of Pharmacy, Tabriz University of Medical Sciences, Tabriz, Iran; ^6^Department of Oral and Maxillofacial Surgery, Faculty of Dentistry, Tabriz University of Medical Sciences, Tabriz, Iran; ^7^Deputy of Food and Drug Administration, Urmia University of Medical Sciences, Urmia, Iran

## Abstract

**Objectives:**

This study presents a discussion on the fundamentals of polymerase chain reaction (PCR) and its use as a diagnostic tool in periodontology.

**Materials and Methods:**

A computer-aided as well as hand-made search in PubMed and Scopus indexed journals (relevant to the topic) was done by keywords of molecular technique in periodontology, PCR, applications of PCR, and PCR in periodontics. Only the papers in the English language and outlining PCR and its association with periodontology were collected and utilized to provide a succinct review. There was no limitation for publication time.

**Results:**

The results of our search showed that PCR has turned into a standard in diagnosis in the field of periodontology. A variety of researches has demonstrated that its sensitive, and specific characteristics make it a quick and effective technique of recognition, identification, and quantification of microorganisms. Identification of various immunoinflammatory markers at the mRNA expression level as well as ascertaining gene-related polymorphisms can also be performed.

**Conclusions:**

The mechanisms of periodontal disease can further become clarified using PCR. *Clinical Relevance*. PCR as a diagnostic method can play a main part in the validation of the clinical diagnosis of periodontal disease indicating the reason, pathogenesis, clinical steps, progress, and prognosis of the disease.

## 1. Introduction

Periodontal disease includes a variety of diseases that are caused by inflammation. If this inflammation is not treated and eliminated, it can cause attachment loss, bone resorption, and eventually tooth extraction [1, 2]. Chronic periodontitis and aggressive periodontitis are two well-known types of soft and hard tissue disease around the teeth that cause the destruction of these tissues [3]. There are two types of classifications for this disease. The first is based on the amount of bone resorption supporting the tooth, divided into localized and generalized. The second is based on the severity of the disease, which in this regard is divided into three categories slight, moderate, and advanced [1, 3, 4]. In the new cataloguing (from 2018), clinical health is also considered, and periodontitis is categorized base on stages, ranging from stage 1 (least severe) to stage 4 (most severe). The risk and rate of disease progression have been categorized into three grades from the lowest risk of progression (grade A) to the highest (grade C). Then, the forms of the disease formerly known as “chronic” or “aggressive” now grouped under a single category, “periodontitis”. The stage-based category is mainly reliant on the severity of disease at appearance as well as on the complexity of disease management. However, the grade-based category offers supplemental data about biological features of the disease [5].

The article "A View on Polymerase Chain Reaction as an Outstanding Molecular Diagnostic Technique in Periodontology" was published in 2021. Journal: Biomed Res Int.

Bacteria in dental plaque cause this chronic disease, and this disease can be seen from the slightest changes in the supporting tissues of the teeth to the severe destruction of the soft and hard tissues supporting the teeth. Bacterial plaques that cause the disease can include bacteria *Porphyromonas gingivalis*, *Aggregatibacter actinomycetemcomitans*, and *Tannerella forsythia*. Still, these are not the only causes of the disease, but the environment and genetics can also predispose people to the disease [6]. As a result, periodontitis is a multifactorial disease, and the presence of pathogenic bacteria in dental plaque cannot cause disease alone. Other factors that help pathogens to cause and promote the disease include an increase in proinflammatory cytokines and a decrease in anti-inflammatory cytokines such as interleukin-10 and the presence of MMP, PGE2, TGF-*β*, and TIMPs [7, 8]. However, evidence suggests that the immune system's response to periodontal disease is much broader.

Measurement of clinical attachment loss (connective tissue attachment loss on the root surface) and radiographic bone loss (alveolar bone loss) is performed for the identification of periodontal diseases in the clinical setting [4, 9]. However, clinical identification of the disease does not determine pathological mechanisms, the way the disease behaves, and advances, and nor does it dictate the prognosis of the disease.

Besides the routine clinical test, diverse techniques of diagnosis are essential in confirmation of the clinical diagnosis. Despite having constitutive benefits, the conventional culture techniques have some disadvantages such as difficult sampling, more time needed for the results, and unable to recognize small quantities of microorganisms [10–13]. Dark field microscopy is incapable of identifying the immobile periodontal pathogens, and flowcytometry, immunofluorescence assay, etc. can yield false-positive results and cross-reactions [14]. Analysis of deoxyribonucleic acid (DNA), ribonucleic acid (RNA), and protein is also performed by the methods in molecular biology. The DNA profiling genetic technique included restriction fragment length polymorphism (RFLP) that made use of diversities in homologous DNA sequences; it is arduous, long in duration, and costly, and a large sample is required. The nucleic acid probe is a nucleic acid molecule that has undergone unnatural synthesis and labeling for the identification of a particular organism accompanied by the restriction of cross-reactivity [14]. Hybridization is defined as the interconnection of complementary DNA strands to create double-stranded nucleic acids and the DNA-DNA hybridization technology with a chequered pattern utilized for epidemiological investigation, and ecologic researches require complicated laboratory equipment and high skills [14].

The article "A View on Polymerase Chain Reaction as an Outstanding Molecular Diagnostic Technique in Periodontology" was published in 2021. Journal: Biomed Res Int.

Polymerase chain reaction (PCR), as a vast diagnostic method, does not have the restrictions stated above and has the capability of recognizing even one copy of the explored DNA targets from clinical microbiologic samples [15–18].

There are complexities in regard to microbiota found in the subgingival area, and utilization of the microbiological methods for the identification and therapeutic management of progressive and resistant forms of periodontitis is dependent upon the diversity of plaque components [19].

A wide variety of advantages in the genetic investigation for research on gene expression has resulted from the evolution of PCR. Identification of the type and frequency of treatment is facilitated by genetic examination utilizing PCR to figure out whether an individual is vulnerable to periodontitis. Precise identification of bacterial strains with divergent phenotype, rapid analysis, ease of quantification, high precision, and least contamination are some main advantages of PCR-based methods. Researches focusing on PCR for assessing mRNA expression of different immune and inflammatory markers are beneficial in recognition of the pathological mechanism of periodontitis.

## 2. Search Methodology

The objective of this review includes a description of the fundamentals, benefits, uses, and restrictions of PCR in periodontology with their future outlooks. A hand-made and computer-aided search in PubMed and Scopus indexed journals pertinent to the topic was done by inputting molecular techniques in periodontology, PCR, applications of PCR, and PCR in periodontics. Sixty-nine articles on the specification of the PCR process along with its association with periodontology were selected to provide a succinct review among 260 articles explored.

The article "A View on Polymerase Chain Reaction as an Outstanding Molecular Diagnostic Technique in Periodontology" was published in 2021. Journal: Biomed Res Int.

## 3. PCR Application in Dentistry

Different types and applications of PCR are summarized in Table 1 and Table 2, respectively. PCR is also of paramount importance in different fields of dentistry. Scraping of the saliva, subgingival plaque, mouthwash, gingival tissue, blood, and buccal mucosa is utilized in PCR for the recognition of microorganisms, mRNA gene expression, and genetic polymorphisms of a diversity of inflammatory mediators in the dental practice [20, 21].

The rapid and sensitive detection of microorganisms in dental plaque samples by the nested PCR method [22], the study of gene expression for the oral anaerobe *P. gingivalis* in periodontal disease *in vivo* by real-time (RT) PCR [23], and examination the expression of the chemokines macrophage inflammatory protein-1 alpha, assay of subgingival overgrowth of pathogenic bacteria in periodontitis by hot-start PCR [24] and interferon-gamma inducible protein 10 and of their respective receptors, CCR5 and CXCR3, by means of reverse transcription-polymerase chain reaction (RT-PCR) techniques [25] have been used in dentistry.

Researches on PCR have well elucidated the knowledge of technology of the oral cavity [49]. Epidemiological researches on the ground of genetic polymorphisms, the microbiology of dental diseases, and their association with systemic diseases may be conducted. PCR is able to recognize pathogens involved in dental caries and describes the pathogenesis of dental caries [50]. Identification of microorganisms involved in endodontic infections is possible [51]. PCR techniques are capable of recognizing genetic markers for oral malignancies and serve as a diagnostic tool as well as aid in treatment prognosis [52].

## 4. PCR Technique in Periodontology

### 4.1. Detection of Microbial Pathogens

The PCR method having more precision, sensitivity, and rapidity is made use of for the recognition and measurement of periodontal bacterial count [19, 53]. Q-PCR or real-time PCR containing primers with specificity in regard to species is able to quantify individual microbial species and total bacterial count in dental plaques precisely [54]. This technique with its precision and sensitivity is a beneficial test for researches on the etiology of periodontal diseases.

The article "A View on Polymerase Chain Reaction as an Outstanding Molecular Diagnostic Technique in Periodontology" was published in 2021. Journal: Biomed Res Int.

Zhou et al. examined the sensitivity and specificity of real-time PCR for periodontal pathogens detection. They used eight periodontal bacteria including *A. actinomycetemcomitans*, *Campylobacter rectus*, *Eikenella corrodens*, *Fusobacterium nucleatum*, *P. gingivalis*, *Prevotella intermedia*, *Streptococcus mutans*, and *T. forsythia* microorganisms. For sensitivity assay, tenfold serial dilution of purified bacterial-specific DNAs was used while specificity assay (specificity of the primer/probe set) was tested by running real-time PCR in parallel against other bacterial-specific DNA. The detection limits of examined bacteria were *S. mutans* 14.31 fg, *P. intermedia* 3.33 fg, *T. forsythia* 0.15 fg, *E. corrodens* 0.40 fg, *F. nucleatum* 0.09 fg, *C. rectus* 1.04 fg, *P. gingivalis* 180 fg, and *A. actinomycetemcomitans* 4.18 fg presenting high sensitivity. No cross-reaction was detected with any of the bacteria, representing high specificity of the method. They concluded that the established test for the quantification of periodontal pathogens using real-time PCR method may be applied in epidemiological assays and as an assistant process for clinical diagnosis of periodontal disease [55].

Numerous periodontal pathogens such as *P. gingivalis*, *A. actinomycetecomitans*, *T. forsythia*, *P. intermedia*, *Prevotella nigrescens*, *Parvimonas micra*, *Capnocytophaga ochracea*, *Capnocytophaga sputigena*, *Eubacteria*, *C. rectus*, and *Capnocytophaga gingivalis* have been recognized in plaque samples found in subgingival areas [56]. The quantity of *P. gingivalis* and *A. actinomycetecomitans* resembled one another in patients with periodontitis as well as control groups, but it was only *A. actinomycetemcomitans*, which was associated with the disease [57]. Identification of *Mycobacterium tuberculosis* in cases where gingiva has increased in size as well cases of osteomyelitis has also been performed by PCR technique [58].

Gram-positive organisms such as *Peptostreptococcus* and *Filifactor*, *Desulfobulbus* and *genera Megasphaera*, classes or phylotypes of *Atopobium*, *Campylobacter*, *Catonella*, *Deferribacteres*, *Dialister*, *Eubacterium*, *Selenomonas*, *Tannerella*, *Streptococcus*, and *Treponema*, the level of which increases in periodontal diseases, have lately been detected by open-ended PCR/sequencing methods [57].

PCR is intended to conduct researches to measure the frequency of herpes simplex virus, human papillomavirus, HIV, human cytomegalovirus, and Epstein-Barr virus type I and II (1 and 2) in the gingival crevicular fluid of patients with different forms of periodontal disease [59, 60]. The use of hot-start PCR was concluded to reveal that the herpes virus might show direct hurt or compromise the resistance of the periodontium to allow subgingival overgrowth of pathogenic bacteria in periodontitis [24].

The article "A View on Polymerase Chain Reaction as an Outstanding Molecular Diagnostic Technique in Periodontology" was published in 2021. Journal: Biomed Res Int.

Evaluation of the microbial extent can be performed following a variety of treatment approaches, thereby making it an index for effective treatment in chronic and aggressive periodontitis [61].

It is also used to examine the relationship of systemic diseases including coronary heart disease, pregnancy complications, diabetes, chronic renal disease, osteoporosis, and respiratory disease with periodontitis by recognizing the quantity of disease-causing agents of the periodontium in different tissue samples such as subgingival plaque, thrombi, carotid endarterectomy, coronary atherosclerotic plaque, aortic valves, placenta, maxillary sinus tissue/wash samples [62, 63].

Diagnostic examinations including the MicroDent® Test, ParoCheck® kits, MyPerioPath® Test, and oral DNA® utilizing multiplex PCR scheme are available on the market for the assessment of microbiota in subgingival plaque samples, and they offer essential details with respect to prevention strategies for healthy individuals and treatment plans for “vulnerable” patients [64].

### 4.2. Detection of Peri-implantitis

PCR has been able to recognize periodontal pathogens such as *A. actinomycetemcomitans*, *P. gingivalis*, *P. intermedia*, *T. forsythensis*, and *Treponema denticola* at peri-implantitis sites [65]. Fungi like *Candida* species were recognized at peri-implantitis and disease-free implant sites and did cocolonization with *P. micra* and *T. forsythia* [66]. The uncultured phyla *Chloroflexi*, *Synergistetes*, and *Tenericutes* and the organisms *P. micra*, *Pseudoramibacter alactolyticus*, *Peptostreptococcus stomatis*, and *Solobacterium moorei* which are linked to peri-implantitis were also recognized [67].

This method is also influential in the recognition of bacteria involved in peri-implantitis prior to loading of implant for the prevention of peri-implantitis [68]. Opportunistic pathogens like *E. faecalis* have been recognized by Q-PCR in the circumference of failed implants recommending removal of the prosthetic appliance and regular disinfection of the implant surface and implant/abutment interface [69].

The positive outcome of dental implant procedures was highly related to a negative TGP (Genetic Test for Periodontitis) specifying polymorphisms of −889 IL1A gene and +3953 IL1B gene utilizing PCR, whereas there existed no relationship between success and a positive result [69].

### 4.3. Detection of Immunoinflammatory Markers

During an imbalance in the oral cavity, the subgingival biofilm stimulates the liberation of proinflammatory cytokines and enzymes originating from the host leading to tissue disintegration. PCR has turned into the standard in protein recognition in periodontic point of view, with microbial antigens, extracellular matrix proteins, and cytokine recognition being of paramount value. The examination of genetic expression of *P. gingivalis* virulence factors was done with the use of Q-PCR [70]. mRNA expression of adhesion molecule (ICAM-1) was determined in *E. corrodens* as a periodontal pathogen that infected epithelial cells using real-time PCR, and it was found to grow in number after being in contact with N-acetyl-D-galactosamine adherence lectin of *E. corrodens* [71].

The article "A View on Polymerase Chain Reaction as an Outstanding Molecular Diagnostic Technique in Periodontology" was published in 2021. Journal: Biomed Res Int.

The ratio was observed to grow using semiquantitative PCR gene expression of receptor activator of NF-KB ligand (RANKL) to osteoprotegerin (OPG) in periodontitis [71].

When Q-PCR was used, there was a relationship between the expression of matrix metalloproteinases and RANKL and the expression of interleukin-1*β*, TNF-*α*, IF-gamma, severe inflammatory reaction, and alveolar bone loss. However, IL-4, IL-10, TIMPs, and OPG expression led a reduction of cellular infiltration and alveolar bone loss [72].

There was a relationship between smoking and mRNA expression of IL-1 *β* with the use of PCR in patients with periodontitis [73]. The expression of specific microRNA species in inflammation of the periodontium targeted and modulated cytokine mRNA using quantitative microRNA PCR assay offers insights to alter periodontal inflammation [74]. Quantitative mRNA expression of different growth factors; toll-like receptors (TLRs), NOD2, and NALP3; and signaling mediators CD14, MYD88, and TIR-domain-containing adapter-producing interferon-beta was also specified by RT-PCR [73].

### 4.4. PCR in Genetic Polymorphism

There is an association between one's vulnerability to periodontitis and genetic factors [75]. The relationship of recognized genetic polymorphisms with phenotypes for particular patient groups currently seems to offer the most inspiring use of genetic factors in the treatment of periodontitis.

Periodontal diseases are influenced by genetic polymorphisms with a number of single-nucleotide polymorphisms (SNPs) taking place in the gene coding for cytokines, receptors, and immune cells linked to the intensity and vulnerability of periodontitis. PCR was utilized for the identification of an altered gene on chromosome 11 which reduced cathepsin C activity leading to Papillon-Lefevre syndrome [76].

PCR has been applied in linkage and segregation analysis of genetic tests in periodontal disease. Various researches have been conducted with the use of PCR investigating the effect of IL-1 gene polymorphism as an intensity determinant on periodontal diseases in a variety of populations and ethnic groups [77].

The article "A View on Polymerase Chain Reaction as an Outstanding Molecular Diagnostic Technique in Periodontology" was published in 2021. Journal: Biomed Res Int.

It was concluded that there was a relationship between TLR-4 gene polymorphism and chronic periodontitis, whereas such a relationship was not found in regard to TLR-9 [78, 79]. Polymorphisms in the Fc gamma receptor gene and MPO-463G/A gene were investigated making use of allele-specific and RT-PCR, respectively, which were concluded to be associated with periodontitis [80]. Other different polymorphisms such as the IL-10 gene, chemokine ligand (CCL5 and CCR5) gene, and OPG gene have been linked to inflammation of the periodontium applying PCR amplification [81, 82].  Table 3 shows the advantages and disadvantages of the PCR method.

## 5. Conclusion and Future Outlooks

The primary step to develop efficacious treatment modalities is the recognition of microbial pathogens correlated to periodontitis. PCR may turn into the optimal recognition tool for disease-causing agents of the periodontium in the near future outstanding to its intrinsic capability of specificity and sensitivity. Examinations of oral diseases can integrate inbred polymorphisms with microbial outlines inside the mouth and might also consist of examines of gene expression and proteomic data calculated in saliva or other oral tissues.

PCR as a vast analytical technique can show a chief share for the validation of the clinical diagnosis of periodontal disease representing the cause, pathogenesis, clinical stages, progress, and prognosis of the disease. As a main example, PCR methods based on amplification of the bacterial gene suggest great applications in clinical samples.

The PCR is an innovator turning point in the arenas of science and medicine, and today, it has turned into a standard analytic and investigation instrument in periodontology. Delving into the pathological mechanisms responsible for the onset, progression, and treatment of the periodontal diseases could remarkably aid in providing active approaches for prevention and treatment in addition to declining the risk issue for pertinent systemic situations. The upcoming of PCR is encouraging in creating more significant understanding beginning from recognition of disease-causing agents of the periodontium to effective treatment approaches. Standardization of the PCR-based methods and their protocols through research laboratories and clinical trials are desired to advance the quality of testified data in the arena of periodontology. Identification of the type and frequency of treatment is facilitated by genetic examination utilizing PCR to figure out whether an individual is vulnerable to periodontitis. The real-time PCR technique is appropriate for microbial examination in individual diagnosis, treatment programs, and control of patients with periodontitis. In-house real-time PCR as an inexpensive technique should be restricted for large studies.

The article "A View on Polymerase Chain Reaction as an Outstanding Molecular Diagnostic Technique in Periodontology" was published in 2021. Journal: Biomed Res Int.

## Figures and Tables

**Table 1:** Different types of PCR techniques.

Different types of PCR techniques	References
Nested PCR	[26]
Multiplex PCR	[27]
Real-time (RT) PCR	[28]
Genomic inverse PCR	[29]
Arbitrary PCR	[30]
Assembly PCR	[31]
Nanoparticle PCR	[32]
Cold-PCR	[33]
Photonic PCR	[34]
Extreme PCR	[35]
Ligation-mediated PCR	[36]
Methylation-specific PCR	[37]
Colony PCR	[38]
Hot start/cold finish PCR	[39]
Core sample PCR	[40]
Dial-out PCR	[39]
Digital PCR	[41]
In silico PCR	[42]
Overlap-extension PCR	[43]
Quantitative PCR	[44]
Solid phase PCR	[45]
Suicide PCR	[46]

**Table 2:** Various applications of the PCR technique (including dentistry applications) [40, 47, 48].

Various applications of the PCR technique
Diagnosis therapy (cancer, diabetes, metabolic, obesity, congenital diseases, neurological disorders, cardiac, etc.)
The ability to amplify RNA
Nucleic acid detection assays
Mycology-parasitology
Clinical bacteriology and virology
Organ transplantation
Agricultural sciences
Studying and understanding the disease state
Dentistry (periodontal diseases, dental caries, oral cancer, and endodontic infections)
Genetic and genomic studies
Insert analysis
Molecular systematic evolution
Tissue typing
Biomarker
Phytopathology
PCR fingerprinting

**Table 3:** Some main advantages and limitations of the PCR technique [48, 83, 84].

*Advantages of PCR*
Precise identification of bacterial strains with divergent phenotype
The ease of quantification
The ability to quantify multiple targets in the clinical specimen
Quality control
Precision
One-minute method for rapid analysis with larger sample size
Rapid analysis
The ability to search for various organisms or genes in one reaction
Least contamination
The study of strictly anaerobic infections
Greater sensitivity
Detection of viruses and mRNA expression levels
Various million times amplification of DNA or RNA
Ability to detect very small amounts of samples
Reproducibility
Facilitating the detection of bacterial DNA present at very low levels
Bacterial identification from bacterial colonies
*Limitations of PCR*
The enormous cost (high test and equipment cost)
Need to achieve high technical skills
Altering the specificity of amplified PCR product
False-positive/False-negative results
There are limitations to creating a high sterile environment
DNA contamination
Low ability to detect between closely related and also highly recombinant species
There are limitations in multiplex PCR mixing different primers
Capable of contaminating other reaction vials

The article "A View on Polymerase Chain Reaction as an Outstanding Molecular Diagnostic Technique in Periodontology" was published in 2021. Journal: Biomed Res Int.

## Data Availability

The raw/processed data required to reproduce these findings can be shared at this time.
